# Interrater and Intrarater Reliability of Electrical Impedance Myography: A Comparison between Large and Small Handheld Electrode Arrays

**DOI:** 10.1155/2021/7296322

**Published:** 2021-11-02

**Authors:** Huijing Hu, Wai Leung Ambrose Lo, Xiaoyun Wang, Le Li, Ping Zhou

**Affiliations:** ^1^Institute of Medical Research, Northwestern Polytechnical University, Xi'an 710072, Shaanxi, China; ^2^Department of Rehabilitation Medicine, The First Affiliated Hospital, Sun Yat-sen University, Guangzhou 510080, Guangdong, China; ^3^Guangdong Work Injury Rehabilitation Center, Guangzhou, Guangdong 510440, China; ^4^University of Health and Rehabilitation Sciences, Qingdao, Shandong 266024, China

## Abstract

The objective of this study was to evaluate the interrater and intrarater reliability of electrical impedance myography (EIM) using handheld sensors of different sizes. Electrical impedance myography of the biceps brachii muscle of twenty healthy individuals was performed by two raters using both large and small sensors. The procedures were also repeated 5 to 8 days after the first recording session. The repeatability of the resistance, reactance, and phase angle at two different current frequencies (50 and 100 kHz) was assessed by the intraclass correlation coefficient (ICC). The ICCs of the large sensor were higher than those of the small sensor for both the intrarater and interrater reliabilities. High-frequency current tended to improve the ICC for the small sensor. These results indicate reasonable repeatability of the handheld electrode arrays for EIM measurements. The findings suggest that electrode array should be selected appropriately according to the size of the tested muscle.

## 1. Introduction

Electrical impedance myography (EIM) is a noninvasive and bioimpedance-based technique that assesses muscle health by applying very low-amplitude (usually a few milliamperes), high-frequency current through a localized area of tissue. It measures the resulting voltage with sensing electrodes on the skin [1]. There are three most commonly used EIM parameters [2], including resistance (*R*), reactance (*X*), and phase angle (*θ*), calculated as *θ* = arctan (X/R). Electrical impedance myography can be used as a biomarker of neuromuscular diseases given that pathological changes (such as muscle atrophy, muscle fiber denervation/reinnervation, and the development of increasing intramuscular fat and connective tissue, etc.) will collectively influence normal impedance characteristics [3]. It has been reported to quantify muscle changes in different neuromuscular diseases, such as amyotrophic lateral sclerosis (ALS), spinal muscular atrophy (SMA), and Duchenne muscular dystrophy (DMD) [4–6]. It has also been used to evaluate paretic muscle changes after neurological injuries [7–9].

Linear EIM involves placement of voltage electrodes along a line over the region of interest, and electrical current is injected far from that region. Previous studies adopted the approach of manually placing the two pairs of electrodes over the skin surface of the tested muscle and reported muscle composition alterations with neuromuscular diseases [4, 5]. This method represents the early stage of EIM and has demonstrated good test-retest reproducibility at 50 kHz [10, 11]. A handheld electrode array (HEA) that has been recently developed provides localized voltage and current electrodes for measuring EIM and has demonstrated very high test-retest reproducibility with multifrequency analysis [12]. Multifrequency EIM is an extension of the linear EIM technique that supplies alternating currents with a range of frequencies rather than just a single frequency. Multifrequency EIM was reported to be more sensitive than single-frequency EIM (50 kHz) in tracking disease progression [13, 14] because multifrequency currents can aid in the extraction of muscle-specific properties (e.g., anisotropy) [15] from the frequency-dependent muscle evaluation.

A gap exists in the field of quantitative measurements of muscle mass, compositional quality, and contractile quality [16], particularly due to the lack of reliable device that can be readily and quickly applied in clinical settings. The EIM assessment procedure involves placing the electrodes on the skin surface. The effects of the skin-electrode interface or the contact sensitivity on bioimpedance outcomes have been a topic of interest [17–19]. Robust EIM measurements can only be obtained via an interface that allows for minor movements without loss of contact; the skin needs to be moist and conductive. Variations in contact levels between raters can result in differences in contact areas, which would reduce the reliability. Geometric factors can also significantly affect measurement reliability, particularly for anisotropic tissues such as skeletal muscles. This is related to the relative direction between the current-injecting electrodes and the underlying muscle fiber orientation. For example, Shiffman found that the muscle impedance was affected by the geometry of the electrode arrangements. The consequences of this entanglement often depend on frequency, making it difficult to extract the properties of the tissue if there are variations in electrode directions among different raters [20]. Particularly, there are different sizes of sensors for measuring EIM, which can affect the relative geometry of the electrode arrangement with respect to the examined muscle. The relative effect of skin and subcutaneous tissues on EIM parameters is also related to sensor size [21]. In addition, the distance between the sensor electrodes can also affect the EIM results. There is gap in the literature in assessing if large or small sensors are sufficiently reliable for clinical application, or if their reliability may differ when measuring a single muscle group by different rates at different time. A recent review by Clark et al. argued that there continues to be a lack of evidence to support the clinical application of EIM in assessing skeletal muscle function [22]. These issues must be addressed to facilitate clinical application of EIM. Therefore, it is critical to evaluate the reliability of EIM measurements and to identify the factors that may affect the EIM outcome via the assessment of between days intrarater and within-day interrater reliability using sensors of different sizes of multifrequency analysis. Motivated by this rationale, the current study assessed the reliability of the two handheld electrode array sensor devices. Intraclass correlation coefficient analysis was conducted to compare the EIM outcomes (*R*, *X*, and *θ*) of the two handheld electrode array sensors, based on the obtained several days apart by the same and different raters. The findings of the study can contribute to our understanding of the reliability of vivo EIM measurement.

## 2. Materials and Methods

### 2.1. Subjects

Healthy individuals were recruited from the student and staff population of the host institute via internal announcement. Included subjects had no reported history of neuromuscular disease. No upper limb weakness or functional impairment was present before or during the data collection period. The study was approved by the Committee for the Protection of Human Subjects (CPHS) of the University of Texas Health Science Center at Houston and TIRR Memorial Hermann Hospital (Houston, TX, USA). The Declaration of Helsinki was strictly followed. All of the subjects were provided with participant information sheet and encouraged to ask questions about the study. Informed written consent was obtained from all of the subjects prior to study enrolment.

### 2.2. Equipment

Impedance measurements were recorded from the biceps brachii muscle of the dominant limb by the HEA system (EIM1103, Skulpt Inc., Boston, MA, USA), which was used in our previous studies [23, 24] A low-intensity electrical current at the frequencies ranging from 1 kHz to 10 MHz was applied in discrete logarithmic steps. The resulting surface voltages were then measured. Two different-sized sensor arrays (Model 20–00036, Small Sensor, and Model 20–0045, Large Sensor) were used in sequence for the repeated measurements. During each measurement, the sensor array was placed over the center of the biceps brachii muscle belly in a longitudinal direction over the muscle fibers. Each sensor contained a pair of current electrodes and a pair of voltage bar electrodes. For the large sensor, the distance between the pair of current electrodes (3.9 cm long; 0.4 cm wide) was 6.8 cm, and the distance between the pair of voltage bar electrodes (1.3 cm long; 0.4 cm wide) was 1.7 cm.  Figure 1(a) shows the configuration of the large sensor. For the small sensor, the distance between the pair of current electrodes (2.6 cm long; 0.2 cm wide) was 3.4 cm, and the distance between the pair of voltage bar electrodes (0.8 cm long; 0.3 cm wide) was 0.8 cm.  Figure 1(b) shows the configuration of the small sensor. Parameters recorded from the wide longitudinal configuration measured along the longitudinal direction were analyzed.

### 2.3. Procedures

The subjects sat on a height-adjustable chair. Their dominant arm rested at 90° flexion and the shoulder at 45° abduction. All data collection took place in the same laboratory. A constant temperature of approximately 22°C was maintained in the laboratory during all data collection sessions. The central air condition system also effectively maintained a stable humidity, although the humidity was not measured. The constant temperature and humidity would ensure similar physical environment for each test session. Each subject was recruited from office work status to participate the study. They were asked not to participate in physical activity on the day before data collection and were given sufficient time to acclimatise to the testing environment upon arrival at the laboratory.

The skin area of the electrode contact was moistened by sterile saline wipes (Hygea, PDI Inc., Hamilton, NY, USA) prior to performing impedance measurements. The HEA was then placed on the muscle until the green “Begin Test” signal was displayed on the computer screen. This indicated good skin contact and ensured the best measurement. Then, data recording was started. During the recording, the device was kept in place until the results were displayed on the screen. The software also plotted the resistance and reactance across the range of frequencies in real time.

Sensors of two different sizes were used in random sequence by each rater. The position of the two array sensors were marked on the skin to minimize confounding factor that was related to site identification between measurements. For intrarater reliability testing, the first rater conducted repeated measurements on two separate occasions with 5 to 8 days apart. Measurements for interrater reliability were collected on the second visit after the first rater completed the measurements.

The assessors received 4 hours of training from a senior technician on the standard operating procedure of the HEA system. This was followed by two hours of unsupervised practice. The associated software was used to visually inspect the data to ensure consistency over three trials.

### 2.4. Parameters

The parameters of resistance (*R*), reactance (*X*), and phase (*θ*) recorded from the longitudinal current electrodes were analyzed. All parameters were obtained at the frequencies of 50 kHz and 100 kHz. These two frequencies were chosen because they were within the optimal range to record EIM responses and were the most commonly used frequencies in previous studies [10, 11].

### 2.5. Data Analysis and Statistics

Statistics analysis was performed using SPSS 23 (IBM Corp., Armonk, NY, USA). The significance level was set at *p* < 0.05. Descriptive analysis was conducted to describe the sample population. The ICC models 2, *k* and 3, *k* were adopted to assess the relative inter-rater and intrarater reliability, respectively. The interpretation of ICC was as follows: ≥0.90 = high reliability, 0.80–0.89 = good reliability, 0.70–0.79 = fair reliability, and ≤0.69 = poor reliability [25]. Absolute reliability indices of standard error of measurements (SEM), smallest real difference (SRD), and Bland–Altman 95% limits of agreement were calculated.

## 3. Results

Twenty healthy participants were recruited (mean age, 32.9 ± 8.2; 12 men and 8 women). A summary of the between-days and within-day longitudinal biceps EIM measurements is shown in Tables 1 and 2. The ICCs of all parameters recorded at 50 kHz and 100 kHz range between 0.90 to 0.98 for the large sensor and between 0.44 and 0.97 for the small sensor. In particular, we note that the ICC value of 50 kHz reactance using the small sensor was 0.440, which indicates poor reliability. The ICCs of the large sensor are higher than the small sensor in all parameters for between-days interrater measurements and within-day measurements. The ICC values recorded by the small sensor at 100 kHz were consistently higher than those recorded at 50 kHz in all parameters, except for reactance, for between-days and within-day measurements. Similar ICC values were observed at the measurements recorded at 50 kHz and 100 kHz by the large sensor. These results indicated that the reliability of the small sensor is prone to be affected by sampling frequency. Tables 3 and 4 present the results of ICC analyses of between-days and within-day measurements recorded by each sensor. Figures 2 and 3 present the ICC plots of longitudinal bicep measurements recorded by the large sensor and small sensor taken by two different raters and by the same rater on different days, respectively.

The SEM and SRD recorded by the large sensor were smaller than those recorded by the small sensor for all measurements, indicating a higher variation around the “true” score and that a larger change is required to be deemed real change. Bland–Altman 95% LOA indicates larger error range between measurements recorded by the small sensor than the large sensor. Tables 3 and 4 present the results of absolute reliability indices for the between-days and within-day measurements recorded by the two assessors using both sensors.

## 4. Discussion

This study aimed to assess the between-day intrarater reliability and within-day interrater reliability of two difference-sized array sensors to record muscle impedance. The results of the present study indicated that the large sensor was consistently more reliable than the small sensor under all tested conditions. The high ICCs are consistent with previous reliability evaluations of localized EIM applications on healthy tibialis anterior muscles [12], as well as in DMD [6, 26]. Rutkove et al. reported high test-retest reliability of linear EIM performed on biceps, quadriceps, and tibialis anterior muscles (ICC = 0.970, 0.971, and 0.938, respectively), 250 days apart at 50 kHz [10].

One of the possible factors that contributes to the lower reliability of the small sensor is the effect of subcutaneous fat over a smaller distance between electrodes. Jafarpoor et al. applied a finite-element model to mimic human upper arm muscles and found that the electrode distance dramatically affected the EIM outputs [27]. All of the tissues beneath the voltage electrodes can in theory contribute to the impedance measurement, including subcutaneous fat and bone. The muscle inherent resistivity is lower than both subcutaneous fat and bones [28]. Therefore, the electrical current tends to pass through the muscle. However, Sung et al. suggested that when currents passed through tissues that were underneath the voltage-measuring electrodes, a considerable proportion of the currents went through the fat at the points closest to where the voltage was recorded [29]. A significant correlation was found between the subcutaneous fat layer (SFL) thickness and the resistance and phase for the medial gastrocnemius muscle in healthy subjects. Jafarpoor et al. also reported that the thickness of the SFL of the quadriceps muscle did contribute to resistance and reactance [27]. Therefore, a shorter electrode distance (small sensor) is more likely to be affected by the SFL than a larger electrode distance (large sensor) [20]. In addition, bioimpedance analysis is influenced not only by the degree of fat mass but also by the electrode-skin interface [19]. The electrode area and distance effects have been evaluated in linear EIM. Rutkove et al. found that a fraction of the effect is related to the electrochemical properties of the electrode-skin-fat-layer complex, whose contribution is inversely proportional to the electrode area [11]. Therefore, the EIM output of the small sensor is more prone to be affected by the electrode-skin-fat-layer than the larger sensor. This in turn may affect the reliability of the small sensor. Findings of this study indicated that EIM measurements should be recorded by electrodes that are properly sized and spaced. Measurement recorded by a relatively small sensor should be considered with caution.

This study observed smaller SEM and SRD recorded by the small sensor at 100 kHz than at 50 kHz, suggesting that the reliability of the instrument is affected by recording frequency. Several studies indicated that multifrequency measures may be more sensitive to disease status and progression over time [13, 14]. By changing the frequency of the current injected, it can shift the relative weights of the resistive (fluid) and reactive (membranes) contributions to the total impedance (i.e., the cell membrane acts like a capacitor in an electrical circuit, such that a very high frequency makes nearly no reactance contribution to the impedance) [30]. At low frequencies, the contact impedance between the sensor and skin is higher, which results in less-reliable data. Hewson et al. studied the impedance of electrode-skin interface using multifrequency (1–16,384 Hz) and found large individual differences in the level of impedance at low frequencies [31]. The findings of this study suggest that higher frequencies (i.e., higher than 50 kHz) should be considered when using the small sensor to record impedance properties.

Reactance has the lowest value of reliability indices among the three EIM parameters recorded by either sensor. Possible contributing factors to the low reactance reliability might be the angle at which the current was applied and the angle measured relative to the muscle fiber direction, and the contact pressure on the skin. There might be small variations in the electrode positions and the angles relative to the biceps brachii each time the electrodes were placed on the skin surface by the rater. The variation in electrode position and the angle relative to biceps brachii may affect the EIM parameters. Tarulli et al. reported that reactance was most sensitive to the angle at which current was applied and the angle measured relative to the muscle fiber direction in bovine skeletal muscles [32]. The sensitivity may be related to the anisotropy of muscle tissue because anisotropy represents the inherent muscle fiber geometry within the muscle, and the electrical currents flow more readily along muscle fibers than passing across them [33]. Therefore, any alteration of the electrode angle affects the direction of injecting currents to the muscle, and in turn, it contributes to the variation of reactance measurements. In addition, reactance is associated with the tendency for oscillating charges to accumulate against the capacitors in the muscle cell membranes [2]. Resistor-capacitor models of the electrode-skin-fat layer interface revealed that the interface resulted in a drift in the EIM results known as the “voltage divider effect,” which depends on the input characteristics of the impedance-measuring instrument, the area, and the conditions of the electrode-skin interface [11]. It can be reduced by increasing the input impedance of the instrument and by using active, low-capacitance probes. Because the measured reactance itself is modeled as a “capacitor,” it is prone to poor contacts between electrode and interface, which in turn can cause the low reliability of reactance.

The limitations of the study should be acknowledged. Although the findings of the current study with healthy population provides useful information about the reliability of small and large EIM sensors, a clinical population was not included in the study while it is important to further extend the reliability investigation to different clinical populations where the EIM can find most important applications. The current study only examined the biceps brachii muscle, although different types of muscles should be further examined. In addition, the same EIM experiment performed by one of the two raters (i.e., the same data set) was used for both the between-days intrarater reliability and within-day interrater reliability investigations. The protocol can be further improved by having both raters take measurements on both days. According to the literature, the variation of muscle size can affect resistance and reactance measurement [29]. For example, the decrease in muscle size might increase measured *R* and *X*. However, the phase angle (*θ*) would be affected to a less extent because its calculation would potentially cancel out simple volumetric effects of the measured muscle [29, 30]. The current study investigated the performance of the large and small sensors over the biceps brachii muscle. It remains a future study to further examine how the EIM parameters change with different muscles.

## 5. Conclusions

EIM measurements of the biceps brachii muscle recorded by the large sensor demonstrated high between-days intrarater and within-day interrater reliability for all three parameters. The small sensor demonstrated poor to high reliability, and repeated measurements were not as consistent as the large sensor. Reactance recorded by the small sensor was the least reliable parameter. The reliability of small sensor was prone to be affected by measuring frequency. Findings of this study suggest that electrode size and interelectrode distance should be selected appropriately in accordance with the size of the tested muscle to achieve the desired reproducibility of EIM measurements.

## Figures and Tables

**Figure 1:** Configuration of electrodes and dimensions of large (a) and small (b) sensors.

**Figure 2:** ICC plots of longitudinal bicep measurements in healthy subjects using large sensors (open triangles) and small sensors (filled circles) taken by two different (inter-) raters. (a) Plots of 50 kHz data. (b) Plots of 100 kHz data.

**Figure 3:** ICC plots of longitudinal bicep measurements in healthy subjects using large sensors (open triangles) and small sensors (filled circles) taken at baseline and 5–8 days later by the same (intra-) rater. (a) Plots of 50 kHz data. (b) Plots of 100 kHz data.

**Table 1:** Between-day longitudinal biceps EIM measurements.

		Large sensor			Small sensor		
		1st measurement	2nd measurement	*d*	1st measurement	2nd measurement	*d*
50 kHz	Phase	20.93(3.52)	21.38 (3.25)	−0.45	12.23 (4.31)	11.75 (3.58)	0.48
	Reactance	9.83 (1.08)	10.13 (1.27)	−0.31	13.31 (3.10)	12.61 (2.72)	0.70
	Resistance	26.59 (6.91)	26.70 (7.16)	−0.11	64.54 (16.60)	63.18 (16.40)	1.36

100 kHz	Phase	22.13 (3.54)	22.56 (3.51)	−0.43	15.17 (3.82)	14.64 (3.27)	0.53
	Reactance	8.46 (1.11)	8.63 (1.31)	−0.17	14.97 (3.16)	14.19 (3.08)	0.77
	Resistance	21.63 (6.38)	21.56 (6.52)	0.07	57.11(15.54)	56.27 (15.53)	0.85

Note: mean (standard deviation); *d*: mean difference between first and second measurements.

**Table 2:** Within-day longitudinal biceps EIM measurements.

		Large sensor			Small sensor		
		1st measurement	2nd measurement	*d*	1st measurement	2nd measurement	*d*
50 kHz	Phase	21.54 (3.34)	21.38 (3.25)	0.15	12.11 (4.07)	11.75 (3.58)	0.36
	Reactance	9.85 (1.16)	10.13 (1.27)	−0.32	12.73 (3.51)	12.61 (2.72)	0.12
	Resistance	25.32 (5.37)	26.70 (7.16)	−1.38	61.67 (7.16)	63.18 (16.39)	−1.38

100 kHz	Phase	22.73 (3.80)	22.56 (3.51)	0.18	14.98 (3.56)	14.64 (3.27)	0.34
	Reactance	8.36 (1.01)	8.63 (1.31)	−0.27	14.14 (3.11)	14.19 (3.08)	−0.05
	Resistance	20.49 (5.04)	21.56 (3.52)	−1.06	54.59 (14.19)	56.27 (15.53)	−1.68

Note: mean (standard deviation); *d*: mean difference between first and second measurements.

**Table 3:** Reliability indices for within-day interrater reliability of both sensors.

Within-day interrater		Large sensor				Small sensor			
		ICC	SEM	SRD	95% LOA	ICC	SEM	SRD	95% LOA
50 kHz	Phase	0.97 (0.92–0.99)	0.19	1.22	−6.38–4.17	0.92 (0.81–0.97)	0.59	2.13	−10.44–6.20
	Reactance	0.90 (0.73–0.96)	0.21	1.27	−4.62–3.29	0.44 (−0.41–0.78)	2.62	4.49	−15.97–8.96
	Resistance	0.99 (0.98–1.00)	0.12	0.96	−7.23–4.59	0.95 (0.88–0.98)	1.53	3.42	−30.09–16.03

100 kHz	Phase	0.98 (0.94–0.99)	0.13	0.99	−5.80–3.88	0.92 (0.81–0.97)	0.51	1.98	−9.41–5.69
	Reactance	0.95 (0.88–0.98)	0.11	0.94	−4.00–2.98	0.67 (0.19–0.87)	1.76	3.68	−14.31–8.13
	Resistance	0.99 (0.98–1.00)	0.11	0.92	−6.34–4.15	0.97 (0.93–0.99)	0.82	2.51	−22.12–12.04

**Table 4:** Reliability indices for between-days intrarater reliability of both sensors.

Between-days intrarater		Large sensor				Small sensor			
		ICC	SEM	SRD	95% LOA	ICC	SEM	SRD	95% LOA
50 kHz	Phase	0.98 (0.95–0.99)	0.13	0.99	−5.66–3.81	0.84 (0.59–0.94)	1.87	3.79	−13.59–7.78
	Reactance	0.90 (0.73–0.96)	0.22	1.30	−4.73–3.35	0.63 (0.02–0.85)	3.30	5.04	−15.28–8.62
	Resistance	0.95 (0.85–0.98)	0.54	2.03	−11.73–6.85	0.95 (0.88–0.98)	2.38	4.27	−29.09–15.52

100 kHz	Phase	0.98 (0.96–0.99)	0.13	1.00	−5.85–3.90	0.91 (0.76–0.96)	0.99	2.76	−10.10–6.30
	Reactance	0.90 (0.74–0.96)	0.22	1.31	−4.76–3.36	0.84 (0.60–0.94)	1.47	3.36	−11.24–6.60
	Resistance	0.96 (0.88–0.98)	0.43	1.81	−10.49–6.22	0.96 (0.89–0.98)	1.98	3.90	−25.98–13.97

## Data Availability

The data sets generated and analyzed during the current study are available from the corresponding author on reasonable request.
